# Ketamine Promotes LPS-Induced Pulmonary Autophagy and Reduces Apoptosis through the AMPK/mTOR Pathway

**DOI:** 10.1155/2022/8713701

**Published:** 2022-07-08

**Authors:** Jianwei Cao, Huiqiang Mai, Yanfen Chen, Ruilin Yuan, Erbin Fang, Meiling Liu, Chunlai Fu

**Affiliations:** ^1^Emergency ICU, The First School of Clinical Medicine, Southern Medical University, Guangzhou, China; ^2^Kangyi VIP Outpatient Clinic, Zhongshan People's Hospital, Zhongshan, China; ^3^Department of Emergency Medicine, Zhongshan People's Hospital, Zhongshan, China; ^4^Department of Pediatrics, Zhongshan Guzhen People's Hospital, Zhongshan, China; ^5^Department of Rehabilitation, Zhongshan Guzhen People's Hospital, Zhongshan, China; ^6^Department of Pediatrics, Zhongshan People's Hospital, Zhongshan, China; ^7^Department of Emergency Intensive Care Unit, Affiliated Dongguan Hospital, Southern Medical University (Dongguan People's Hospital), Dongguan, China

## Abstract

To explore the protective effect of ketamine on acute lung injury (ALI) in sepsis mice regarding the autophagy and apoptosis, lipopolysaccharide (LPS) was used to construct a sepsis-induced ALI model. In *in vivo* experiments, ketamine at a concentration of 20 mg/kg was injected before modeling. The serum levels of inflammatory factors IL-1*β*, IL-6, and TNF-*α* were detected by enzyme-linked immunosorbent assay (ELISA) kit. At the same time, quantitative real-time polymerase chain reaction (qRT-PCR) was used to detect apoptosis-related factors Bax and Bcl-2 and autophagy-related factors Beclin-1 and P62. In *in vitro* experiment, firstly, Cell Counting Kit-8 (CCK8) assay was used to detect the cell viability and identify optimal concentration of ketamine. TUNEL staining, Western blotting (WB), and qRT-PCR were used to detect alveolar type II epithelial cells (AEC II) AEC II cell apoptosis. The content of inflammatory factors in the cell supernatant was detected by kits and the autophagy intensity of AEC II cells was detected by PCR and WB. At the same time, the expression changes of AMPK/mTOR pathway were detected by WB technology. Compared with the Sham group, the dry-wet ratio of the lung tissue in the LPS group was obviously increased, the expression of inflammatory factors in the serum was upregulated, and apoptosis and autophagy activation occurred. In the LPS + ketamine group, ketamine significantly promoted autophagy intensity and inhibited inflammatory response, thereby reducing apoptosis. *In vitro*, 1 mmol/L ketamine can effectively improve the viability of AEC II cells after LPS treatment, promote autophagy, and decrease cell apoptosis. And we found that the above-mentioned effect of ketamine was by regulating the activation of AMPK/mTOR pathway. In this study, we demonstrated that LPS treatment can induce inflammation and autophagy and induce apoptosis in lung cells. In contrast, AMPK expression was activated after ketamine treatment, inhibiting the mTOR pathway and promoting autophagy, thereby alleviating the apoptosis of AEC II cells.

## 1. Introduction

Sepsis refers to the systemic inflammatory response caused by infection [1]. The clinical manifestations range from fever and rapid heart rate to dyspnea, decreased blood pressure, confusion, oliguria, and other organ dysfunctions. Sepsis is the leading cause of death in critically ill patients in the intensive care unit. Even after timely anti-infection and supportive treatment, the mortality rate is still as high as 20%–60% [2, 3]. In the United States, there are 750,000 patients with sepsis each year, and 215,000 of them die of sepsis. Even with this calculation, the annual incidence of sepsis in our country has reached 3 million, and nearly one million people die from sepsis every year [4, 5]. The main cause of death in sepsis is multiple organ dysfunction syndrome (MODS) caused by infection, among which ALI or acute respiratory distress syndrome (ARDS) is the most common. After nearly decades of research, although the research on the diagnosis and treatment of the pathogenesis of ALI has made great progress, so far no specific drugs have been found to treat ALI [6].

Autophagy is a behavior in which cells degrade various macromolecular substances and damage organelles through lysosomes. In recent years, the role of autophagy in regulating inflammation and apoptosis in the host has not been fully elucidated, but it is clear that autophagy can affect the progression and prognosis of inflammatory diseases [7]. In the pathogenesis of ALI caused by sepsis, the intensity of autophagy in alveolar epithelial cells and the uncontrolled release of inflammatory mediators are the important reasons leading to the lung injury of sepsis. Therefore, it is still crucial to further explore the regulatory mechanism of autophagy in sepsis-induced ALI [8].

As an intravenous anesthetic, ketamine has analgesic, sedative, and anti-inflammatory effects. At present, the anti-inflammatory effect of ketamine has been confirmed by a large number of studies. Ketamine can inhibit the inflammatory response of various inflammatory cells such as macrophages, neutrophils, and monocytes [9]. Recent studies have found that the anti-inflammatory effect of ketamine is related to the inhibition of autophagy. In a mouse model of cerebral ischemia-reperfusion (I/R) injury, ketamine can activate mTOR to reduce the inflammatory response of cerebral I/R [10]. Therefore, the mechanism of using ketamine to regulate autophagy will provide an idea for the development of new drugs and new therapies for the treatment of ALI caused by sepsis.

Studies have found that, in inflammatory diseases, AMPK, an AMP-dependent protein kinase, an important upstream of autophagy, is activated. At the same time, the autophagy process is regulated by the mTOR signaling pathway, and mTOR can sense changes in cell nutrients and metabolism. Activated mTOR will promote the synthesis of mTORC1 and mTORC2 protein complex, thereby inhibiting autophagy [11]. As mTOR is a key factor in autophagy regulation, whether the anti-inflammatory effect of ketamine is related to the activation of mTOR and downregulation of autophagy remains to be confirmed.

## 2. Materials and Method

### 2.1. Animal

Thirty SPF-grade C57BL/6 male mice aged 8 weeks weighing 18–22 g were purchased from the Experimental Animal Center of Southern Medical University; the mice were kept in breeding cages, 5 mice per cage. All mice were raised in the laboratory of the animal center of our hospital. Mice were housed in a temperature controlled room (21 ± 2°C) on a 12 : 12 h light/dark cycle (lights on at 06:00). All mice had free access to water and food. This study was approved by the Animal Ethics Committee of Southern Medical University Animal Center.

### 2.2. Sepsis Induced ALI Model

The ALI mice model was established based on a previous study [12]. Firstly, the mice were anesthetized by intraperitoneal injection of 1% sodium pentobarbital 5–6 ml/kg, the mice were fixed on the operating table with tape, and the whole layer of skin was cut in turn from the middle of the neck with tissue scissors, neck muscles, and muscles. The membrane was fully separated to expose the trachea. Next, a syringe was used to pierce the airway, and 4 ml/kg LPS (Tianpu Biochemical Pharmaceutical, Guangzhou, China) was instilled; then the mouse was upright for a few minutes to fully absorb LPS. Finally, the full-thickness skin of the mouse was sutured with 3-0 stitches. Mice in the ketamine-treated group were injected intramuscularly with ketamine at a concentration of 20 mg/kg (Tianpu Biochemical Pharmaceutical, Guangzhou, China) 30 minutes before the model preparation, and the Sham group and the model group were injected with the same amount of normal saline. Blood was taken 6 hours after the operation, and lung tissues were quickly cut out, placed in liquid nitrogen for quick freezing, and then stored at −80°C.

### 2.3. Lung Dry-Wet Ratio Measurement

We isolated the lung tissues 6 hours after the ALI model and then stored it in a 60°C oven for continuous uninterrupted baking for 48–72 hours. After the baking, the dry weight of the lung tissue was determined on an electronic scale. The value of wet weight/dry weight was the lung dry-wet ratio.

### 2.4. Enzyme-Linked Immunosorbent Assay (ELISA) to Detect Serum Inflammatory Factors

After drawing blood from the mice heart, the serum was separated and then centrifugated at a speed of 3000 rpm for 10 minutes at 4°C. The lower layer of blood cell pellet wad discarded, while the upper layer of serum was absorbed. Serum protein sample was added to each well, followed by being shaken in a shaker at room temperature for 2 hours. After being washed with phosphate buffered saline (PBS), 100 *μ*L conjugate was added to each well for incubation for 2 hours. The substrate working solution was configured according to the kit instructions (Thermo Fisher Scientific, Waltham, MA, USA) and then added to each well for incubation for 30 minutes in the dark. Finally, the optical density (OD) value of each well at 450 nm was detected with a microplate reader, and the protein concentration of each sample was calculated according to the standard curve.

### 2.5. Cell Culture and Processing

The culture of alveolar type II epithelial cells (AEC II) used Dulbecco's Modified Eagle's Medium (DMEM; Life Technology, Wuhan, China; containing 10% fetal bovine serum (FBS, Life Technology, Wuhan, China), 1% penicillin, and streptomycin) to culture the cells, and we placed them in an incubator at 37°C and 5% CO_2_. In the experiment, we pretreated AEC II cells with 1 mmol/L ketamine for 6 hours and then treated the cells with LPS for 6 hours as the time point for the study.

### 2.6. Cytometric Bead Array (CBA) Detects Cell Supernatant Inflammatory Factors

According to the kit instructions (Construction, Nanjing, China), after constructing the cytokine standard solution, the supernatant was added to the standard solution and incubated for 2 hours at room temperature in the dark. Next, the washing solution was used to wash the beads and added to the 96-well plate, followed by incubation at room temperature for 2 hours. Finally, after washing the beads again with the washing solution, the signal intensity was measured by flow cytometry.

### 2.7. Cell Counting Kit-8 (CCK8) Assay Detects Cell Viability

According to the correct operation of the kit instructions (Camilo Biological, Nanjing, China), 3000 cells per well were seeded in a 96-well plate, and the models of each group were replicated after the cells adhered. The prepared CCK-8 mixture was added to the sample wells, and the 96-well plates were incubated in an incubator for 2 hours. Then, a microplate reader was used to measure the absorbance of each well at 450 nm.

### 2.8. Western Blotting Technology

After washing the sample three times with a precooled PBS buffer, the protein lysate was used to ice lyse the cells for 30 minutes. After full lysis, the suspension was centrifuged, and the supernatant was collected. Then the bicinchoninic acid (BCA, Construction, Nanjing, China) kit was used to measure the protein concentration, and the protein was denatured at high temperature. Sodium dodecyl sulfate-polyacrylamide gel electrophoresis was carried out sequentially. After the polyvinylidene difluoride (PVDF, Thermo Fisher Scientific, Waltham, MA, USA) membrane was transferred, it was blocked with 10% skim milk for 2 hours, then combined with the primary antibody (P62, Abcam, Cambridge, MA, USA, Rabbit, 1 : 2000; Beclin-1, Abcam, Cambridge, MA, USA, Rabbit, 1 : 3000; Bcl-2, Abcam, Cambridge, MA, USA, Mouse, 1 : 2000; Bax, Abcam, Cambridge, MA, USA, Mouse, 1 : 2000; AMPK, Abcam, Cambridge, MA, USA, Rabbit, 1 : 2000; mTOR, Abcam, Cambridge, MA, USA, Rabbit, 1 : 2000; p-mTOR, Abcam, Cambridge, MA, USA, Rabbit, 1 : 5000; GAPDH, Proteintech, Rosemont, IL, USA, 1 : 5000), and incubated overnight at 4°C. The next day, the membranes were incubated with the second antibody for 1 hour, followed by being washed with tris buffered saline-tween (TBST) 3 times. Then, electrochemiluminescence (ECL) luminescent solution (Yifei Xue Biotechnology, Nanjing, China) was added in the dark room and incubated for 1 minute. The fluorescence chemiluminescence imaging system was used for photography. Meanwhile, Quantity One software was used to analyze the gray value of the strip.

### 2.9. Quantitative Real-Time Polymerase Chain Reaction (qRT-PCR)

Total RNA was extracted with TRIzol (Thermo Fisher Scientific, Waltham, MA, USA) method. RNA concentration was measured by spectrophotometer and reverse-transcribed into complementary deoxyribose nucleic acid (cDNA) in turn. Then PCR amplification was performed under the below conditions: 10 min denaturation at 95°C; 40 cycles of denaturation at 95°C for 15 s; 60°C annealing for 30 s; and 72°C extension for 30 s. The comparative threshold cycle (Ct) method, that is, the 2^−ΔΔCt^ method, was used to calculate fold amplification [13]. The primer sequences are shown in Table 1.

### 2.10. TUNEL Staining

Strictly operate according to the instructions of the Terminal Deoxynucleotidyl Transferase dUTP Nick End Labeling (TUNEL) staining kit (Elabscience, Wuhan, China). After mounting the slides with anti-fluorescence quencher containing 4′,6-diamidino-2-phenylindole (DAPI), we observed it under a fluorescence microscope. Each group of cells randomly selected 3 high-power (×200) fields to calculate the AEC II cell apoptosis rate. Apoptosis rate = TUNEL positive cells/100 × 100%. We took the average percentage of 3 visual fields as the result, and the experiment was repeated three times.

### 2.11. Statistical Analysis

Using Statistical Product and Service Solutions (SPSS) 20.0 statistical software analysis (IBM, Armonk, NY, USA), all measurement data are expressed as mean ± standard deviation (mean ± SD), single-factor analysis of variance is used between groups of samples in multiple groups, Least Significant Difference (LSD) is used for pairwise comparison, and *P* < 0.05 is considered statistically significant.

## 3. Results

### 3.1. LPS Treatment Induced Acute Lung Injury in Mice

We collected lung tissues and serum at the sixth hour after LPS treatment and weighed the wet weight of fresh lung tissue and then baked the lung tissue in a 60°C oven for 48 hours-72 hours and then weighed the dry weight to calculate the lung dry-wet weight ratio. It was found that the ratio of the ALI group was obviously greater than that of the Sham group, indicating that after LPS-induced ALI, pulmonary edema was obviously worse than that of the Sham group. Conversely, the dry-wet weight ratio of the ALI + ketamine group was obviously lower than that of the ALI group (Figure 1(a)). Secondly, ELISA kits were used to detect the expression of IL-1*β*, IL-6, and TNF-*α* in serum. The results showed that the expression of IL-1*β*, IL-6, and TNF-*α* in the ALI group was obviously higher than that in the Sham group, while the expression of the above-mentioned inflammatory factors in the ketamine treatment group was obviously reduced (Figures 1(b)–1(d)). Next, we used qRT-PCR to detect apoptosis and autophagy-related molecules in lung tissue. The results showed that the expression of Bax and Beclin-1 mRNA in the ALI group was obviously increased, while the expression of Bcl-2 and P62 mRNA was obviously decreased. However, in the ALI + ketamine group, we found that the mRNA expressions of Bax and P62 were lower than those of the ALI group, while the mRNA expressions of Bcl-2 and Beclin-1 were higher than those of the ALI group. qRT-PCR results showed that LPS could promote apoptosis and autophagy in lung tissue, but ketamine treatment could further promote autophagy and alleviate apoptosis (Figures 1(e) and 1(f)).

### 3.2. Apoptosis Increased after LPS Treatment of AEC II Cells

In order to further clarify the apoptosis effect of LPS on ALI, we selected AEC II cells as the research object. First, the CCK8 assay was used to explore the optimal processing concentration of ketamine. The results showed that when AEC II cells treated with LPS were cultured with 1 mmol/L ketamine, the cell viability was highest (Figure 2(a)). Next, in order to clarify the anti-apoptotic effect of ketamine, we used TUNEL staining to detect the apoptosis rate of AEC II cells. As shown in Figure 2(b), the TUNEL positive ACEII cells in the LPS group was obviously increased, while rate in the LPS + ketamine group decreased. qRT-PCR detection of Bax and Bcl-2 also found that the expression of Bax mRNA in the LPS group increased, while the expression of Bcl-2 mRNA decreased (Figure 2(c)). At the same time, WB also obtained similar results (Figure 2(d)).

### 3.3. Increased Inflammation and Autophagy Intensity after LPS Treatment of AEC II Cells

Then, by detecting the expression of IL-1*β*, IL-6, and TNF-*α* in the cell supernatant, it was found that the expression of IL-1*β*, IL-6, and TNF-*α* in the LPS group was increased, while the expression in the LPS + ketamine group was obviously decreased (Figures 3(a)–3(c)). qRT-PCR detection of Beclin-1 and P62 mRNA expression showed that LPS could promote Beclin-1 expression in AEC II cells and reduce the expression of P62, while ketamine can further promote Beclin-1 expression and inhibit P62 expression in AEC II cells (Figure 3(d)). In addition, the results obtained by WB were similar to the former (Figure 3(e)).

### 3.4. Ketamine Inhibits LPS-Induced AMPK Pathway Activation

AMPK/mTOR pathway has been found in numerous articles to regulate autophagy and apoptosis. Therefore, we used WB experiments to detect the expression of this pathway in cells. WB results showed that, after LPS treatment, AMPK expression increased, while p-mTOR expression decreased. What is interesting is that in the LPS + ketamine group the expression of AMPK was still increased, and the expression of p-mTOR was obviously suppressed, but there was no significant difference in the expression of mTOR among the three groups. Meanwhile, the p-mTOR/mTOR ratio in the LPS + ketamine group was lower than that in the LPS group and control group (Figure 4).

## 4. Discussion

In this study, we chose C56BL/6 mice as the research object of the animal experiment. LPS was instilled into the trachea to construct a sepsis-induced ALI mouse model. Six hours after instillation of LPS, the mice developed symptoms of respiratory distress such as shortness of breath. Arterial blood gas analysis showed that the oxygenation index PaO2/FiO < 300 mmHg, which met the clinical diagnostic criteria of ARDS, namely, ALI [14]. At the same time, in *in vitro* experiments, we used LPS to treat AEC II cells to construct an ALI model, because AEC II are essential for the study of lung development, damage, and repair, and AEC II cells are essential for the study of ALI-related diseases.

After organ injury, the main change in cytology is cell death, which is also one of the important pathological changes in sepsis. The latest research found that, in addition to cell necrosis and apoptosis, another method of cell death-autophagy has also been discovered [15]. Autophagy is originally meant to engulf itself, has a high degree of species homology, is widely present in eukaryotic cells, and has the functions of degradation of error proteins, phagocytosis of bacteria, and antigen presentation [16]. Therefore, we can focus on autophagy as a research target and expand new prospects for the treatment of ALI caused by sepsis by regulating autophagy. In the sepsis model, after LPS stimulation and bacterial infection, autophagy increases, which can play a role in protecting cells and reducing cell death [17]; as in this experiment, autophagy expression was upregulated after LPS treatment. At the same time, autophagy in the state of starvation or inflammation, autophagic vesicles can provide nutrients by degrading intracellular components and reduce cell damage, but if this state continues for too long, it will cause excessive consumption of cells and lead to autophagic cells death [18]. In this experiment, we have also verified that after LPS treatment the cell inflammatory response was obvious, and the expression of apoptosis-related molecules and the apoptosis rate in AEC II cells were obviously increased. After treatment with ketamine, the degree of autophagy was increased, while inflammation and apoptosis were reduced. Therefore, we speculated that ketamine can reduce cell damage by promoting the intensity of autophagy.

At present, the role of AMPK/mTOR pathway in inflammation, autophagy, and apoptosis has been extensively studied. Studies have shown that inhibiting the expression of mTOR phosphorylation can reduce the number of inflammatory cells, thereby achieving anti-inflammatory effects [19]. However, in our study, p-mTOR decreased after LPS treatment, but inflammatory factors did not. This may be because the LPS-induced autophagy intensity was insufficient to eliminate too many inflammatory factors, while ketamine could further inhibit the phosphorylation expression of mTOR, promote autophagy intensity, and thus play a role in inhibiting inflammation. Therefore, we hypothesized that the intensity of autophagy determines the different effects on the inflammatory response and the degree of apoptosis.

## 5. Conclusions

In this study, we confirmed that, whether *in vivo* or *in vitro*, LPS treatment induces inflammation and autophagy in lung cells, leading to apoptosis. In contrast, AMPK expression was increased after ketamine treatment, and the mTOR pathway was inhibited to promote autophagy, thereby improving apoptosis of AEC II cells. This will provide a new research mechanism for the treatment of sepsis-induced ALI.

## Figures and Tables

**Figure 1:** LPS treatment induced acute lung injury in mice. (a) The dry-wet weight ratio of the ALI + ketamine group was obviously lower than that of the ALI group. (b)–(d) ELISA assay was used to detect changes in IL-1*β*, IL-6 and TNF-*α* in lung tissues. Ketamine significantly reduced the levels of IL-1*β*, IL-6 and TNF-*α*. (e) and (f) qRT-PCR was used to detect changes in Bax, Bcl-2, Beclin-1 and p62 expression levels in lung tissues. Results showed that mRNA expressions of Bax and P62 were lower than those of the ALI group, while the mRNA expressions of Bcl-2 and Beclin-1 were higher than those of the ALI group. (“^*∗*^” indicates that compared with the Sham group, “#” indicates that compared with ALI group *P* < 0.05).

**Figure 2:** Apoptosis increased after LPS treatment of AEC II cells. (a) CCK8 assay was used to detect the AEC II cell viability. Cell viability significantly increased after treatment with 1 mmol/L ketamine. (b) TUNEL staining was used to detect the AEC II apoptosis rate, and statistical analysis of the positive rate. The TUNEL positive ACEII cells in the LPS group was obviously increased, while rate in the LPS + ketamine group decreased. (c) qRT-PCR was used to detect mRNA changes in Bax and Bcl-2 expression levels in AEC II cells. Ketamine increased mRNA expression of Bcl-2, while reduced Bax level. (d) WB was used to detect protein changes in Bax and Bcl-2 expression levels in AEC II cells and gray value analysis. Ketamine increased protein level of Bcl-2, while reduced Bax. (“^*∗*^” indicates that compared with the Control group, “#” indicates that compared with LPS group *P* < 0.05).

**Figure 3:** Increased inflammation and autophagy intensity after LPS treatment of AEC II cells. (a)–(c) ELISA assay was used to detect changes in IL-1*β*, IL-6 and TNF-*α* in supernatant. The expression of IL-1*β*, IL-6 and TNF-*α* in the LPS group was increased, while the expression in the LPS + ketamine group was obviously decreased. (d) qRT-PCR was used to detect mRNA changes in Beclin-1 and p62 expression levels in AEC II cells. Ketamine increased Beclin-1 mRNA expression and inhibited P62 mRNA expression in AEC II cells. (e) WB was used to detect protein changes in Beclin-1 and p62 expression levels in AEC II cells and gray value analysis. Ketamine increased Beclin-1 protein expression and inhibited P62 protein expression in AEC II cells. (“^*∗*^” indicates that compared with the Control group, “#” indicates that compared with LPS group *P* < 0.05).

**Figure 4:** Ketamine inhibits LPS-induced AMPK pathway activation. Wsetern blot was used to detect protein changes in AMPK, mTOR and p-mTOR expression levels in AEC II cells and gray value. The p-mTOR/mTOR ratio in the LPS + ketamine group was significantly lower than that in the LPS group (“^*∗*^” indicates that compared with the Control group, “#” indicates that compared with LPS group *P* < 0.05) analysis.

**Table 1:** Real time PCR primers.

Gene name	Forward (5′ > 3′)	Reverse (5′ > 3′)
Beclin-1	ATGGAGGGGTCTAAGGCGTC	TCCTCTCCTGAGTTAGCCTCT
P62	AGGATGGGGACTTGGTTGC	TCACAGATCACATTGGGGTGC
BAX	CAGTTGAAGTTGCCATCAGC	CAGTTGAAGTTACCATCAGC
Bcl-2	GACTGAGTACCTGAACCGGCATC	CTGAGCAGCGTCTTCAGAGACA
GAPDH	ACAACTTTGGTATCGTGGAAGG	GCCATCACGCCACAGTTTC

RT-PCR, quantitative real-time polymerase chain reaction.

## Data Availability

The datasets used and analyzed during the current study are available from the corresponding author on reasonable request.

## References

[1] Cecconi M., Evans L., Levy M., Rhodes A. (2018). Sepsis and septic shock. *The Lancet*.

[2] Faix J. D. (2013). Biomarkers of sepsis. *Critical Reviews in Clinical Laboratory Sciences*.

[3] Rello J., Valenzuela-Sánchez F., Ruiz-Rodriguez M., Moyano S. (2017). Sepsis: a review of advances in management. *Advances in Therapy*.

[4] Rowe T. A., McKoy J. M. (2017). Sepsis in older adults. *Infectious Disease Clinics of North America*.

[5] Berg D., Gerlach H. (2018). Recent advances in understanding and managing sepsis. *F1000Research*.

[6] Mo Y., Lou Y., Zhang A. (2018). PICK1 deficiency induces autophagy dysfunction via lysosomal impairment and amplifies sepsis-induced acute lung injury. *Mediators of Inflammation*.

[7] Glick D., Barth S., Macleod K. F. (2010). Autophagy: cellular and molecular mechanisms. *The Journal of Pathology*.

[8] Zhao H., Chen H., Xiaoyin M. (2019). Autophagy activation improves lung injury and inflammation in sepsis. *Inflammation*.

[9] Chang E. I., Zarate M. A., Arndt T. J. (2018). Ketamine reduces inflammation pathways in the hypothalamus and Hippocampus following transient hypoxia in the late-gestation fetal sheep. *Frontiers in Physiology*.

[10] Wang C.-Q., Ye Y., Chen F. (2017). Posttraumatic administration of a sub-anesthetic dose of ketamine exerts neuroprotection via attenuating inflammation and autophagy. *Neuroscience*.

[11] Zhang X., Zheng J., Yan Y. (2019). Angiotensin-converting enzyme 2 regulates autophagy in acute lung injury through AMPK/mTOR signaling. *Archives of Biochemistry and Biophysics*.

[12] Matute-Bello G., Frevert C. W., Martin T. R. (2008). Animal models of acute lung injury. *American Journal of Physiology - Lung Cellular and Molecular Physiology*.

[13] Zhou J., Xu J., Sun S., Guo M., Li P., Cheng A. (2021). N-acetylcysteine slows down cardiac pathological remodeling by inhibiting cardiac fibroblast proliferation and collagen synthesis. *Disease Markers*.

[14] Rice T. W., Wheeler A. P., Bernard G. R., Hayden D. L., Schoenfeld D. A., Ware L. B. (2007). Comparison of the s 2 ratio and the Pa o 2/F io 2 ratio in patients with acute lung injury or ARDS. *Chest*.

[15] D’Arcy M. S. (2019). Cell death: a review of the major forms of apoptosis, necrosis and autophagy. *Cell Biology International*.

[16] Saha S., Panigrahi D. P., Patil S., Bhutia S. K. (2018). Autophagy in health and disease: a comprehensive review. *Biomedicine & Pharmacotherapy*.

[17] Qiu P., Liu Y., Zhang J. (2019). Review: the role and mechanisms of macrophage autophagy in sepsis. *Inflammation*.

[18] Matsuzawa-Ishimoto Y., Hwang S., Cadwell K. (2018). Autophagy and inflammation. *Annual Review of Immunology*.

[19] Mushaben E. M., Kramer E. L., Brandt E. B., Khurana Hershey G. K., Le Cras T. D. (2011). Rapamycin attenuates airway hyperreactivity, goblet cells, and IgE in experimental allergic asthma. *The Journal of Immunology*.

